# Breast Tumor Classification Using Intratumoral Quantitative Ultrasound Descriptors

**DOI:** 10.1155/2022/1633858

**Published:** 2022-03-07

**Authors:** Sabiq Muhtadi

**Affiliations:** Department of Electrical and Electronic Engineering, Islamic University of Technology, Gazipur, Bangladesh

## Abstract

Breast cancer is a global epidemic, responsible for one of the highest mortality rates among women. Ultrasound imaging is becoming a popular tool for breast cancer screening, and quantitative ultrasound (QUS) techniques are being increasingly applied by researchers in an attempt to characterize breast tissue. Several different quantitative descriptors for breast cancer have been explored by researchers. This study proposes a breast tumor classification system using the three major types of intratumoral QUS descriptors which can be extracted from ultrasound radiofrequency (RF) data: spectral features, envelope statistics features, and texture features. A total of 16 features were extracted from ultrasound RF data across two different datasets, of which one is balanced and the other is severely imbalanced. The balanced dataset contains RF data of 100 patients with breast tumors, of which 48 are benign and 52 are malignant. The imbalanced dataset contains RF data of 130 patients with breast tumors, of which 104 are benign and 26 are malignant. Holdout validation was used to split the balanced dataset into 60% training and 40% testing sets. Feature selection was applied on the training set to identify the most relevant subset for the classification of benign and malignant breast tumors, and the performance of the features was evaluated on the test set. A maximum classification accuracy of 95% and an area under the receiver operating characteristic curve (AUC) of 0.968 was obtained on the test set. The performance of the identified relevant features was further validated on the imbalanced dataset, where a hybrid resampling strategy was firstly utilized to create an optimal balance between benign and malignant samples. A maximum classification accuracy of 93.01%, sensitivity of 94.62%, specificity of 91.4%, and AUC of 0.966 were obtained. The results indicate that the identified features are able to distinguish between benign and malignant breast lesions very effectively, and the combination of the features identified in this research has the potential to be a significant tool in the noninvasive rapid and accurate diagnosis of breast cancer.

## 1. Introduction

According to the World Health Organization (WHO) factsheet, breast cancer is the world's most prevalent form of cancer, with a staggering 7.8 million patients being diagnosed in the 5-year period between 2016 and 2020 [1]. It was the most commonly diagnosed form of cancer, as well as the second leading cause of cancer-related deaths for women in 2020 [2]. Early diagnosis of breast cancer is crucial to the survival of patients due to its role in treatment selection as well as prediction of response to therapy [3].

Ultrasound imaging has established itself as an important noninvasive screening technique for breast cancer [4]. It retains a significant advantage over other modalities such as mammography due to its nonionizing nature, low costs, and high portability. Furthermore, ultrasound imaging can improve tumor detection during breast cancer diagnosis by as much as 17% [5], as well as reduce the number of nonessential biopsies by 40% [6]. However, ultrasound imaging suffers from system and operator dependency [7, 8] which negates its reproducibility. Furthermore, conventional ultrasound imaging procedures are qualitative in nature, and thus radiological evaluation of ultrasound B-mode images relies heavily on the diagnostic experience of the radiologist.

Quantitative ultrasound (QUS) techniques represent a domain of ultrasound imaging procedures which extract various quantitative measures of tissue microstructure [9, 10]. Unlike conventional ultrasound imaging techniques, QUS procedures are independent of the system and operator related factors [11, 12] and as a result are highly reproducible. Furthermore, QUS techniques can provide an indication of diagnosis without the need for expert evaluation and thus have the potential for rapid diagnosis of conditions such as breast cancer. The utility of QUS techniques has been established over multiple areas, such as differentiation between benign and malignant thyroid tissues [13], detection of prostate cancer [14, 15], and characterization of carotid plaques [16]. Several different quantitative parameters have also been explored by researchers with regard to characterization of breast tissue.

QUS spectroscopy involves extraction of spectral parameters from the attenuation-corrected normalized power spectrum of raw ultrasonic radiofrequency signals. Lizzi et al. [17, 18] proposed the linear parameterization of this normalized power spectrum in order to extract the spectral slope, spectral intercept, and midband fit of ultrasound echoes. These features provide a measure of shape, size, concentration, and power of acoustic scatterers and have been applied for both diagnosis of breast lesions [19, 20], as well as noninvasive evaluation of response to chemotherapy [21, 22] with notable success.

The statistics of the acquired ultrasound envelope signal can be modelled as a probability density function (PDF) in order to analyze the scattering properties of soft tissue. Several well-known statistical distributions may be utilized in this regard to model the statistics of the envelope, and two popular distributions which are applied to model scattered signals from the breast are the Nakagami and homodyned K distribution. The Nakagami distribution was proposed for the modelling of ultrasonic backscatter by Shankar [23]. Several approaches have been proposed by researchers for the classification of breast lesions using the characteristics of the Nakagami distribution. The parameters of the distribution have been analyzed for their potential as quantitative descriptors of breast cancer by themselves [24], through compounding approaches [25], in conjunction with the parameters of other distributions such as the K distribution [26], as well as in conjunction with other types of quantitative descriptors such as entropy and texture [27, 28]. The homodyned K distribution was proposed for the modelling of ultrasound echoes by Dutt and Greenleaf [29] and later modified by Hruska [30] and Hruska and Oelze [31]. The homodyned K distribution parameters have been applied in conjunction with breast imaging reporting and data system (BIRADS) descriptors as well as shear wave elasticity (SWE) features for the classification of breast lesions [32, 33].

Tumors are known to exhibit heterogeneities in physiology, microenvironment, and metabolism, which is significant for the characterization of cancer [34–37]. These heterogeneities may be quantified using texture analysis techniques [38]. In the context of ultrasonic B-mode images, texture analysis provides an indication of gray-level transitions by analyzing the spatial relationships between neighboring pixels in an image, and this is useful for evaluating the differing textures exhibited by benign and malignant masses [20]. With this rationale, texture analysis techniques applied to ultrasound scans have been utilized by several studies for the characterization of breast lesions [39–42].

This study proposes a breast tumor classification system that utilizes the three major types of QUS features used by researchers to characterize breast lesions: spectral features, envelope statistics features, and texture features. To my knowledge, no other research works have evaluated the features analyzed in this study simultaneously for breast cancer diagnosis. A total of 16 different features were extracted from ultrasound patient data for evaluation across two different datasets, of which one is balanced, and the other is severely imbalanced. Holdout validation was used to split the balanced dataset into 60% training and 40% testing sets, and feature selection in the form of sequential forward selection (SFS) was applied to the training set to identify the subset of features most relevant to the classification of benign and malignant breast tumors. The performance of the identified features was evaluated on the test set, where a maximum classification accuracy of 95% and an area under the receiver operating characteristics curve (AUC) of 0.968 were obtained. The performance of the identified relevant features was further validated on the imbalanced dataset, where a hybrid resampling strategy was firstly utilized to create an optimal balance between benign and malignant samples. A maximum classification accuracy of 93.01%, sensitivity of 94.62%, specificity of 91.4%, and AUC of 0.966 were obtained. The results indicate that the identified features are able to distinguish between benign and malignant breast lesions very effectively, and the combination of the features identified in this research work has the potential to be a significant tool in the noninvasive rapid and accurate diagnosis of breast cancer.

## 2. Materials and Methods

### 2.1. Description of Datasets

#### 2.1.1. OASBUD Dataset

The Open Access Series of Breast Ultrasonic Data (OASBUD) [43] was utilized in this study. It consists of ultrasound radiofrequency (RF) data of 100 breast lesions of patients at the Oncology Institute in Warsaw. Among these, 52 were malignant lesions, and 48 were benign. All malignant lesions were histologically assessed by core needle biopsy. 37 out of the 48 benign lesions were also histologically assessed; the remaining 13 did not qualify for a biopsy but were observed by a radiologist over a 2-year period. The ultrasound data was recorded at the Department of Ultrasound, Institute of Fundamental Technological Research Polish Academy of Sciences, and the study was approved by the Institutional Review Board (IRB). Patients were examined by a radiologist with 18 years of experience, following the BI-RADS guidelines as well as the Polish Ultrasound Society standards. For each lesion, two individual longitudinal and transverse scans were recorded using an Ultrasonix SonixTouch Research ultrasound scanner with an L14-5/38 linear array transducer and a center frequency of 10 MHz. Each scan consisted of 512 RF lines, and the signals were digitized using a 40 MHz sampling frequency. The region of interest (ROI) for each individual scan was indicated by the radiologist.

#### 2.1.2. ATL Dataset

The ultrasound data from ATL's premarket approval (PMA) IRB-approved study undertaken in 1994 [19] was also used for this research. It consists of ultrasound RF data of breast lesions from 130 patients. Among these, 104 were benign and 26 were malignant, all histologically assessed by core needle biopsy. The ultrasonic data was recorded at three clinical sites, Thomas Jefferson University, University of Cincinnati, and Yale University, during routine ultrasonic examinations of patients scheduled for biopsy. The tumors were examined by an experienced radiologist using a Phillips Ultrasound UM-9 HDI scanner, with an L10-5 linear array transducer and a center frequency of 7.5 MHz. The L10-5 transducer was used at a default power level and a single transmit focal length, as selected by the operator. All standard ultrasonic breast examination procedures were maintained during the examination. Multiple views were selected by the radiologist for every lesion, which included at least a radial and an antiradial view. The signals were digitized by interfacing a Spectrasonics Inc. (King of Prussia, PA) acquisition module using a 20 MHz sampling frequency and an effective dynamic range of 14 bits. Time-gain-control (TGC) data was obtained before each scan, and the acquired data was corrected for TGC before processing. As can be observed, the dataset contains quite a high imbalance ratio between benign and malignant cases (4 : 1).

### 2.2. Feature Extraction

Three types of features were extracted from patient ultrasound scans for use in this study: spectral features, envelope statistics features, and texture features. All processing codes were written in MATLAB™ (The MathWorks, Inc., Natick, MA).

#### 2.2.1. Spectral Features

Spectral features were obtained from parametric images formed using spectrum analysis parameters [18, 44, 45]. A Hamming window of length 2.4 mm was applied to the RF data of each ultrasound patient scan. The power spectrum of the windowed RF data was then computed using the Fourier transform and expressed in dB. Linear regression was applied to the power spectrum over the 6 dB bandwidth of the signal. This regression analysis yields the slope (SL) of the regression line, the value at midpoint (MBF) of signal bandwidth, and the intercept at zero frequency (INT). Images of these parameters were formed by progressively sliding the Hamming window over each RF data with an overlap of 87.5% and repeating the above sequence.

The linear regression line which approximates the normalized power spectrum can be expressed as

(1) $$\begin{array}{c} P\left(f\right)=I+sf, \end{array}$$

where *f*, *s*, and *I* represent frequency, SL, and INT, respectively. Thus, the MBF can be expressed as

(2) $$\begin{array}{c} M=I+sf_{0}, \end{array}$$

with *f*_0_ representing center frequency of the usable bandwidth.

The presence of frequency-dependent attenuation affects the MBF and SL values obtained during analysis [19]. To compensate for this, the attenuation (in dB) is assumed to vary linearly with frequency, and this approximation is validated through the findings of Alam et al. [19] and Bamber [46] on the invariance of intercept in the presence of attenuation. For this study, the MBF and SL were corrected as follows:

(3) $$\begin{array}{c} M_{\alpha }=P_{\alpha }\left(f_{0}\right)=I-\left(s-2\alpha d\right)\;f_{0}, \end{array}$$

(4) $$\begin{array}{c} s_{\alpha }=\left(s-2\alpha d\right), \end{array}$$

where *α* represents the effective attenuation coefficient and *d* represents the depth of the intervening tissue. The value of the attenuation coefficient *α* was set to 1.0 dB/MHz-cm, based on the attenuation coefficient for muscle reported by Mast [47].

Figure 1 illustrates the three types of spectral parametric images (MBF, INT, and SL) that are formed from ultrasound RF data. The mean and standard deviation of pixel values from the intratumoral region of these parametric images were used in this study for the classification of breast cancer.

#### 2.2.2. Envelope Statistics Features

Ultrasonic pulses moving through tissue are subject to scattering due to artifacts located within the tissue, which are aptly termed as “scatterers.” Consequently, the backscattered ultrasonic echo signal received at the transducer can be viewed as the superposition of scattered signals from individual scatterers within the tissue [48]. Application of a statistical distribution model to this backscattered ultrasound envelope can provide information related to tissue microstructure. Two such statistical distribution models that effectively describe the scattering characterization of ultrasound echo signals from breast tissue are the Nakagami distribution [23] and the homodyned K distribution [31].

*(1) Homodyned K Distribution*. The homodyned K distribution is an analytically complex model; however, it is more versatile than models such as the Rayleigh distribution and the K distribution [49]. The probability density function (pdf) *H*(*A*) of the homodyned K distribution is expressed in the form of an improper integral [29] as follows

(5) $$\begin{array}{c} H\left(A\right)=A\;\int_{0}^{\infty }xJ_{0}\left(sx\right)\;J_{0}\left(Ax\right){\left(1+\frac{x^{2}\sigma^{2}}{2\mu }\right)}^{-\mu }dx\;, \end{array}$$

where *J*_0_ is a zero-order Bessel function of the first kind, *s*^2^ is the coherent signal energy, *σ*^2^ is the diffuse signal energy, and *μ* is a measure of the effective number of scatterers in the target cell. The ratio of the coherent to diffuse signal can be used as a derived parameter *k* = *s*/*σ* to define the periodicity in scatterer locations. The parameters *k* and *μ* are believed to provide an accurate description of tissue scattering properties [49].

The homodyned K parameter estimation technique outlined by Hruska et al. [31] was utilized for this study. This technique uses the signal-to-noise ratio (SNR), skewness, and kurtosis of fractional order moments to estimate the parameters of the homodyned K distribution.

A third parameter, the diffuse-to-total signal power ratio [50] *h* = 1/(*k* + 1), is also defined. The parameters *μ*, *k*, and *h* were estimated by fitting the homodyned K distribution to all samples within the tumor region of each ultrasound envelope image, and these parameters were then utilized for the classification of breast lesions.

*(2) Nakagami Distribution*. The Nakagami distribution [51] was introduced by Nakagami (1943, 1960) in the context of wave propagation. It is far less analytically complex than the homodyned K distribution. The pdf *N*(*A*) of the ultrasonic backscattered envelope under the Nakagami distribution model is given by

(6) $$\begin{array}{c} N\left(A\right)=\frac{2m^{m}A^{2m-1}}{\Gamma \left(m\right)\Omega^{m}}e^{-\frac{{mA}^{2}}{\Omega }}U\left(A\right). \end{array}$$

Here, Γ(.) and *U*(.) represent the Euler gamma function and the unit step function, respectively.

The Nakagami distribution has two parameters, expressed as follows:

(7) $$\begin{array}{c} m=\frac{{\left[E\left(R^{2}\right)\right]}^{2}}{E{\left[R^{2}-E\left(R^{2}\right)\right]}^{2}}, \end{array}$$

(8) $$\begin{array}{c} \Omega =E\left[R^{2}\right], \end{array}$$

where *R* represents the ultrasonic backscattered envelope and *m* is referred to as the shape parameter, providing information about envelope statistics. In the case of the Nakagami distribution, it is constrained such that *m* ≥ 0.5 [51], in which case it is referred to as the Nakagami parameter. *Ω* is a scaling parameter.

The similarity between the Nakagami distribution and the K distribution may be used to define a third parameter of the Nakagami distribution. The K distribution has a cumulative distribution expressed as

(9) $$\begin{array}{c} F_{K}\left(r\right)=\frac{2b}{\Gamma \left(M\right)}\;{\left(\frac{br}{2}\right)}^{M}K_{M-1}\left(br\right)r\geq 0\;M\geq 0, \end{array}$$

where *M* provides a measure of the effective number of scatterers in the target cell and *b* is a scaling parameter. The parameters of the K distribution can be expressed in terms of the Nakagami distribution [24]:

(10) $$\begin{array}{c} M=\frac{2m}{1-m}, \end{array}$$

(11) $$\begin{array}{c} b=2\sqrt{\frac{2m}{\Omega \left(1-m\right)}}. \end{array}$$

Using this relationship, a parameter *α* can be defined, where *α* = 1/*b*, or

(12) $$\begin{array}{c} \alpha =\frac{1}{2}\sqrt{\frac{\Omega \left(1-m\right)}{2m}}, \end{array}$$

where *α* is defined as the effective cross-section of scatterers in the target cell [24].

The parameters *m*, *Ω*, and *α* were estimated by fitting the Nakagami distribution to all samples within the tumor region of the ultrasound envelope image, and these parameters were then utilized for the classification of breast lesions.

#### 2.2.3. Texture Features

The texture of the ultrasound envelope images was quantified using gray-level cooccurrence matrix (GLCM) techniques. GLCM techniques quantify texture by evaluating the spatial relationship between neighboring pixels in an image [41]. A GLCM matrix is created by calculating how often a pixel with gray-level intensity value *i* occurs adjacent to a pixel with the value *j*. Let *P*(*i*, *j*) denote the GLCM matrix representing the probability of having neighboring pixels with gray-level intensities *i* and *j* in the ultrasound image. Let *μ* and *σ* denote the mean and standard deviation for row *i* or column *j* of the GLCM matrix. The following four parameters may be defined from such a matrix

(13) $$\begin{array}{c} \text{Contrast}=\underset{i,j}{\sum }{\left|i-j\right|}^{2}P\left(i,j\right), \end{array}$$

(14) $$\begin{array}{c} \text{Correlation}=\frac{1}{\sigma_{i}\sigma_{j}}\underset{i,j}{\sum }\left(i-\mu_{i}\right)\left(j-\mu_{j}\right)P\left(i,j\right), \end{array}$$

(15) $$\begin{array}{c} \text{Energy}=\underset{i,j}{\sum }P^{2}\left(i,j\right), \end{array}$$

(16) $$\begin{array}{c} \text{Homogeneity}=\underset{i,j}{\sum }\frac{P\left(i,j\right)}{1+\left|i-j\right|}. \end{array}$$

Contrast represents a measure of gray-level variations in the parametric image. Correlation provides an indication of the linear correlation between neighboring pixels. Energy quantifies textural uniformity between neighboring pixels, and homogeneity represents a measure of the incidence of pixel pairs of different intensity within the parametric image. To extract GLCM features, an ROI composed of the minimum bounding rectangular area around the tumor of each ultrasound envelope image was formed, similar to the procedure followed by [41]. The full range of gray levels in each ROI was linearly scaled into 16 discrete gray levels. GLCM matrices were then formed at five interpixel distances, 1, 2, 3, 4, and 5 pixels, and at four angular directions, 0°, 45°, 90°, and 135°, and the four GLCM features were calculated from each of the GLCM matrices. All four texture features were averaged over distances and angular directions to obtain final values for each patient and then used for classification of breast lesions.

### 2.3. Resampling of ATL Dataset

As noted before, the ATL dataset contains a high level of imbalance between benign and malignant cases (4 : 1). A hybrid resampling strategy is applied in order to mitigate the imbalance between the classes. The number of majority class instances are firstly reduced using undersampling to decrease the imbalance ratio between classes. Oversampling is then performed to generate new minority class samples in order to balance the dataset. The hybrid strategy creates an optimal balance between the classes and ensures the quality of the resampled data. Synthetic minority oversampling (SMOTE) [52] is used for oversampling, while Tomek links [53] are used for undersampling. They are described below.

#### 2.3.1. Smote

SMOTE is an oversampling technique that is used to synthesize minority class instances based on their nearest neighbors and is frequently applied to address class imbalance in the medical domain [54]. Consider an *k*-dimensional dataset with samples of *x*_*i*_, where *x*_*i*_ = (*i* = 1, 2, 3, ⋯..*n*) and *k* represents the number of features. Let *A* represent the majority class with *c* samples and *B* represent the minority class with *d* samples, such that *c* + *d* = *n* and *c* ≥ *d*. SMOTE processes the dataset as follows: (i) for each minority class sample *b*_*i*_ (*i* = 1, 2, ⋯, *d*) , identify its *T* nearest neighbors, (ii) select a sample *b*_*j*_ from the *T* nearest neighbors of *b*_*i*_ and generate a synthetic data sample *p*_*i*_ = *x*_*i*_ + (*x*_*j*_ − *x*_*i*_) × *λ*, where *λ* *ϵ* [0, 1] is a random number, (iii) repeat *s*_*i*_ times to obtain *s*_*i*_ new synthetic samples of *b*_*i*_. In this work, a *T* value of 5 was used.

#### 2.3.2. Tomek Links

Tomek link is an undersampling method that is used to eliminate majority instances from the dataset whenever a “Tomek link” is found. Let *b*_*i*_ denote a sample from the minority class and *a*_*i*_ denote a sample from the majority class. Then *b*_*i*_ and *a*_*i*_ are said to form a Tomek link pair if there is no sample *x*_*k*_ such that *d*(*b*_*i*_, *x*_*k*_) < *d*(*b*_*i*_, *a*_*i*_), where *d* is used to represent distance between two samples. In this instance, the majority sample *a*_*i*_ is eliminated as a process of under sampling.

### 2.4. Sequential Forward Selection

Sequential forward selection (SFS) is a wrapper method that adds relevant features to the selected feature subset over multiple iterations on the basis of an evaluation criterion. The process begins with an empty subset of selected features. In the first iteration the model is trained using each feature individually, and the best performing feature is identified based on the evaluation metric and added to the selected feature subset. In the second iteration, the model is trained using pairings of the already selected feature along with each of the remaining features. The performance of each pair is analyzed using the evaluation metric, and the feature that achieves the best performance when paired with the first feature is added to the selected feature subset, but only if the performance of the pair is higher than the performance of the best individual feature in terms of the evaluation criterion. This process is repeated over multiple iterations until no improvement in the evaluation criterion is obtained by adding more features. The misclassification rate was used as the evaluation criterion in this study.  Figure 2 illustrates a flowchart of the SFS process.

### 2.5. Performance Evaluation

A total of 16 features were extracted from the intratumoral region of ultrasound scans in both OASBUD and ATL datasets: (i) mean of MBF, (ii) standard deviation of MBF, (iii) mean of INT, (iv) standard deviation of INT, (v) mean of SL, (vi) standard deviation of SL, (vii) *k* (homodyned K), (viii) *μ* (homodyned K), (ix) *h* (homodyned K), (x) *m* (Nakagami), (xi) *Ω* (Nakagami), (xii) *α* (Nakagami), (xiii) contrast, (xiv) correlation, (xv) energy, and (xvi) homogeneity. Most lesions in both datasets were scanned at multiple intersecting scan planes, thereby providing complementary data for a given lesion. If a lesion had multiple scans, each quantitative feature value for multiple scans of a specific lesion was averaged to arrive at a single number. A two-sided Wilcoxon rank sum test (95% confidence) was performed on each of the extracted features in both datasets to assess statistical significance between benign and malignant groups. The purpose of the statistical test was solely to demonstrate discrimination capability of the extracted features.

The OASBUD dataset was used to determine the relevant features for classification of breast lesions as it contains a healthy balance between benign and malignant cases. Holdout validation was utilized to split the OASBUD dataset into 60% training and 40% testing sets. SFS was applied on the training set to identify the best performing features, and the performance of these features was evaluated using the test set. Three different algorithms were used for classification: (i) K-nearest neighbor (KNN) with Mahalanobis distance and a K value of 5, (ii) support vector machine with linear kernel (SVM), and (iii) random forest (RF). KNN predicts the class of an unknown data sample based on the class of the “K” nearest samples through a majority voting scheme. SVM identifies a linear hyperplane in the feature space that maximizes the margin between the classes and distinctly classifies the data samples. RF is a robust bagging algorithm that uses an ensemble of decision trees to classify random subsets of the training samples and makes a final classification prediction through majority voting.

The ATL dataset was used to validate the performance of the identified relevant features and ensure transferability. Due to limited number of samples, the ATL dataset could not be used as a completely independent test set. However, both 10-fold stratified cross-validation (SCV) and leave-one-out cross-validation (LOOCV) were utilized to evaluate the performance of the features on the ATL dataset, as both of these methods are appropriate for performance evaluation of smaller datasets. Furthermore, the ATL dataset contains a high imbalance ratio (4 : 1 between negative and positive samples). To mitigate this, SMOTE and hybrid SMOTE-Tomek resampling techniques were applied on the ATL dataset, and the performance of the features with and without sampling was analyzed. SMOTE by itself increased the number of positive (malignant) samples from 26 to 104, to provide a completely balanced scenario. Meanwhile, the SMOTE-Tomek procedure reduced the number of negative samples (benign) from 104 to 93 and increased the number of positive samples from 26 to 93, again providing a completely balanced scenario.

Classification results are evaluated by analyzing the receiver operating characteristic (ROC) curve, in particular the area under the curve (AUC), sensitivity, specificity, and accuracy. AUC is a single scalar value which ranges between 0 and 1 (1 indicating significant performance) representing the predictive performance of a classification task. Accuracy is the ratio of the total number of correct predictions to the total number of instances in a classification task. Sensitivity is a measure of correctly classified positive instances (malignant cases), and specificity is a measure of correctly classified negative instances (benign cases). MATLAB™ (The MathWorks, Inc., Natick, MA) was used to develop all models and evaluate all performance metrics.

## 3. Results

Table 1 denotes the mean and standard deviation of all features in the OASBUD dataset for benign and malignant cases, as well as the *p* value and level of statistical significance of the features. Statistical significance is divided into three levels based on *p* value: not statistically significant (*p* ≥ 0.05) indicated by “~,” statistically significant (*p* < 0.05) indicated by “∗,” and extremely significant (*p* < 0.001) indicated by “∗∗.” Table 2 similarly denotes mean and standard deviation feature values for benign and malignant cases in the ATL dataset, as well as statistical significance of the features.

SFS applied on the training split of the OASBUD dataset identified 4 out of the 16 features as the most significant to breast cancer diagnosis:

- *k* (homodyned K)
- *h* (homodyned K)
- *m* (Nakagami)
- *Ω* (Nakagami)

Figure 3 illustrates the representative box and scatter plots of these four features from the OASBUD dataset.

Table 3 denotes the performance parameters obtained by the three classifiers on the testing portion of the OASBUD dataset using the 4 selected features.  Figure 4 illustrates the ROC curves obtained by the three classifiers.

Figure 5 illustrates the representative box and scatter plots of the four selected features from the ATL dataset.

Table 4 denotes the performance parameters obtained by the three classifiers on the unsampled ATL data using the 4 selected features with both 10-fold SCV and LOOCV.  Table 5 provides the performance parameters for the ATL dataset after SMOTE was applied, and Table 6 provides the performance parameters after hybrid SMOTE-Tomek was applied.

Figure 6 illustrates the ROC curves obtained by the three classifiers on the unsampled and resampled instances of the ATL dataset using both validation schemes.

## 4. Discussion

This study proposes a breast tumor classification system using the three major types of intratumoral QUS descriptors. A total of 16 different QUS parameters are extracted from the intratumoral region of breast ultrasound RF scans, consisting of spectral features, envelope statistics features, and texture features. Sequential forward selection was utilized to identify the most relevant subset of features for breast cancer diagnosis.

Analyzing the statistical significance of each of the 16 features extracted from the OASBUD dataset (Table 1), it can be clearly seen that the envelope statistics features (homodyned K features: *k*, *μ*, and *h* and Nakagami features: *m*, *Ω*, and *α*) are more statistically significant than spectral features or texture features for distinguishing between benign and malignant samples. A similar scenario is observed in Table 2, where the envelope statistics features were found to be more statistically significant than the other types of extracted features for the ATL dataset.

The OASBUD dataset was used to identify the most relevant QUS features for the classification of breast lesions, as the proportion of positive and negative classes is similar. Using a balanced dataset enables feature selection techniques to identify key features that can distinguish between the positive and negative class effectively without bias towards any specific class. All four features selected by the SFS algorithm were related to envelope statistics. Thus, the feature selection algorithm seems to be selecting the most statistically relevant features for breast cancer diagnosis. Specifically, two features were chosen from the homodyned K distribution, and two features were chosen from the Nakagami distribution. Thus, a significant finding of this study is that envelope statistics features are able to segregate between breast lesion types more effectively than the spectral and texture features analyzed in this study. A hypothesis for this may be the fact that envelope statistics are able to describe the subresolutional properties of tissue better than spectral analysis and provide more distinguishing capability than features obtained from analyzing the spatial relationships between pixels in ultrasound envelope images.

Analyzing the performance parameters obtained on the testing portion of the OASBUD dataset using the four selected features (Table 3), it can be observed that all three classifiers obtained similar AUC of around 0.96. In terms of classification accuracy, sensitivity, and specificity, the SVM classifier obtained slightly lower performance than the KNN or RF classifiers. The best performance was clearly obtained using the RF classifier, with a classification accuracy of 95%, sensitivity of 95%, and specificity of 95%.

The ATL dataset was used to validate the performance of the identified relevant features. However, due to the limited number of samples in this study, the ATL dataset could not be used as an independent test set to classify models trained only by the OASBUD dataset. Two validation schemes were utilized to demonstrate that the performance does not suffer from any bias. Both 10-fold SCV and LOOCV are established validation schemes for validation of smaller datasets.

As mentioned before, the ATL dataset contains a high imbalance ratio between positive and negative cases. The impact of this can be observed from the performance parameters provided in Table 4. All three classifiers inadvertently became biased towards the negative class (which represented the majority), as observable by the very low sensitivity values and very high specificity values. For both 10-fold SCV and LOOCV, the KNN classifier provided the poorest performance. The best performance was obtained by the RF classifier using 10-fold SCV, with a moderate sensitivity of 65.38%, accuracy of 85.38%, and AUC of 0.8711.

Application of SMOTE introduced a large number of synthesized positive samples (representing the minority class). This significantly improved performance, particularly in terms of sensitivity (Table 5). The KNN classifier and the RF classifier obtained the highest sensitivity using 10-fold SCV: 94.23% and 92.31%, respectively. However, there was a disparity between the sensitivity and specificity values in these two cases, with both classifiers also correspondingly obtaining lower specificity measures. Thus, applying SMOTE by itself may introduce bias towards the positive minority class, particularly for highly imbalanced cases such as the ATL dataset where a large number of samples need to be synthesized.

To account for this, a hybrid SMOTE-Tomek procedure is utilized, which firstly reduces majority class instances to decrease the imbalance ratio between the classes and then performs oversampling. This approach ensures quality of resampled data, as the number of samples needed to be synthesized is lower. Analyzing Table 6, it can be observed that the disparity between sensitivity and specificity is much lower than those obtained in Table 5, particularly for the two cases discussed above. The best performance was obtained by the RF classifier, with a classification accuracy of 93.01%, sensitivity of 94.62%, specificity of 91.4%, and AUC of 0.9660 obtained using 10-fold SCV and classification accuracy of 91.4%, sensitivity of 93.55%, specificity of 89.25%, and AUC of 0.9640 obtained using LOOCV. Both cases represent significant performance for breast tumor characterization. The results obtained are compared with two recent multiparametric QUS studies for breast cancer in Table 7.

It should be noted that the procedure for acquisition of envelope statistics features differed in this work from other literature. In general, envelope statistics features are estimated by fitting the statistical distribution (i.e., Nakagami or homodyned K) at several small windows spanning the ROI [27, 28, 33]. Following this, the statistical parameters for each distribution (i.e., Nakagami *m*, Nakagami *α*, and homodyned *k*) are estimated at each window, and the final feature value is taken as the average parameter value across all the windows [27, 28, 33]. This methodology reduces impact of signal attenuation at different depths. However, in this study, rather than using windows, the statistical distribution model (both Nakagami and homodyned K) was fit on all samples within the tumor region, and the envelope statistics features were acquired correspondingly from this. This methodology was chosen at it fits the distribution model on a larger pool of samples (i.e., all the samples within the tumor), which ensures a more stable estimation of the statistical parameter for each distribution. However, it does not take into account signal attenuation like the methodology discussed previously, and future studies may analyze the impact of this on breast tumor characterization.

This study has a few limitations. Firstly, it utilizes a limited amount of patient data. Ideally, such a study should utilize a large pool of ultrasound RF data, apply feature selection on a large training set, and validate performance on a significant testing set. Although two datasets were utilized in this study, they were not mixed. The two datasets were acquired at a difference of about 20 years, and thus, the quality of ultrasound signals in the OASBUD dataset should be far superior to those present in the ATL dataset. This may be a likely cause for the difference in feature values for the two datasets (Tables 1 and 2). Furthermore, a concern with the ATL dataset is the sampling frequency utilized during data collection. Generally, sampling frequency is chosen to be about 4 times higher than the transducer central frequency [56]. The 20 MHz sampling frequency used for a transducer central frequency of 7.5 MHz may lead to loss of information. It should be noted that this condition was met in case of the OASBUD dataset, which used a 40 MHz sampling frequency for a transducer central frequency of 10 MHz. Thus, rather than combining the two datasets physically, the datasets were combined artificially, where the recently acquired OASBUD dataset was used to identify relevant features, and the ATL dataset was used to validate the performance of the identified features. Another limitation of this study is the large imbalance present in the ATL dataset, which necessitates the application of resampling techniques. In an ideal scenario, sampling should not be applied to the test set, as the characteristics of the test set should coincide with medical data available in the real world where imbalance is very prevalent. However, without sampling, the classifiers used in this research become very strongly biased towards the positive majority class and provide poor sensitivity as highlighted in Table 4. This is unacceptable, as correctly identifying malignant cases is of crucial importance. The resampling techniques used in this paper were intended to display that, in a case where the positive and negative classes are fairly balanced, the identified features will be able to distinguish between benign and malignant lesions very effectively. This objective is achieved considering the significant improvement in performance, particularly in terms of sensitivity, after resampling techniques were used to balance the ATL dataset (Tables 5 and 6). Another issue is the undersampling approach that was utilized. The Tomek link technique removes benign samples in the feature space that are close to malignant samples, which may inevitably translate to overly optimistic results. However, in this study, Tomek links was not applied on the ATL dataset by itself, but rather as part of the hybrid SMOTE-Tomek strategy. The purpose of Tomek links in this framework was to act as a data cleaning method and remove overlapping samples created after application of SMOTE, rather than simply removing benign samples that were originally present in the dataset. Such techniques are commonly utilized after application of SMOTE in order to prevent overgeneralization. Next, the spectrum of ultrasonic signals acquired during evaluation of spectral features are not only dependent on tissue properties but also on the two-way transfer function of the transducer and the ultrasonic module (system effects), the beam properties corresponding to the two-way range dependent diffraction function (diffraction effects) and acoustic attenuation [23]. As most lesions analyzed in this study lie at similar depths (2-3 cm), system and diffraction effects will not significantly affect the acquired spectrum analysis parameters, and hence, these effects were not accounted for in this study. However, acoustic attenuation was considered, as it is known to significantly affect SL and MBF values obtained from ultrasound images [23]. Furthermore, this study opted sequential forward selection (SFS) to identify the most relevant texture features, as it is a relatively simple wrapper technique which has been shown to be very effective [57]. Future studies may analyze more robust selection algorithms such as fuzzy rough set-based selection procedures [58] or ensemble selection approaches [59].

## 5. Conclusion

This study proposes a breast lesion classification system using the three major types of intratumoral QUS descriptors that can be extracted from ultrasound radiofrequency (RF) data. A total of 16 QUS features corresponding to spectral features, envelope statistics features, and textural features were extracted from ultrasound patient data. Four features from envelope statistics were identified as the most significant by feature selection. These four features were able to distinguish between tumor types with a high level of accuracy across two datasets. This demonstrates the capability of the identified features in characterization of benign and malignant breast lesions, and the combination of features identified in this research work has the potential to aid the diagnostic procedure associated with noninvasive screening and diagnosis of breast tumors. The scope of this study can be further enhanced by incorporating more advanced feature selection procedures, incorporating more patient data, and including other types of features in the analysis, for instance more advanced texture features obtained from gray-level run length matrix (GLRLM) and gray-level size zone matrix (GLSZM) techniques, as well as statistical features such as information entropy.

## Figures and Tables

**Figure 1:** (a) Ultrasound B-mode image and corresponding (b) midband fit (MBF) parametric image, (c) spectral intercept (INT) parametric image, and (d) spectral slope (SL) parametric image.

**Figure 2:** Flowchart of sequential forward selection (SFS) algorithm.

**Figure 3:** Box and scatter plots of (a) *k* (homodyned K), (b) *h* (homodyned K), (c) *m* (Nakagami), and (d) *Ω* (Nakagami) values from the OASBUD dataset.

**Figure 4:** ROC curves obtained by the three classifiers using the 4 selected features in the testing portion of the OASBUD dataset.

**Figure 5:** Box and scatter plots of (a) *k* (homodyned K), (b) *h* (homodyned K), (c) *m* (Nakagami), and (d) *Ω* (Nakagami) values from the ATL dataset.

**Figure 6:** ROC curves obtained by the three classifiers using the 4 selected features in (a) unsampled ATL data with 10-fold SCV, (b) unsampled ATL data with LOOCV, (c) ATL data with SMOTE applied and 10-fold SCV, (d) ATL data with SMOTE applied and LOOCV, (e) ATL data with hybrid SMOTE-Tomek applied and 10-fold SCV, and (f) ATL data with hybrid SMOTE-Tomek applied and LOOCV.

**Table 1:** Feature values for benign and malignant cases and statistical significance of features in the OASBUD dataset.

Feature	Benign values	Malignant values	*p* value	Statistical significance
Mean of MBF	88.25 ± 6.84	92.06 ± 9.25	<0.05	∗
Standard deviation of MBF	4.61 ± 0.86	5.08 ± 1.19	<0.05	∗
Mean of INT	95.19 ± 4.25	91.8 ± 6.56	<0.05	∗
Standard deviation of INT	14.98 ± 0.78	15.32 ± 0.76	<0.05	∗
Mean of SL	−4.54 ± 0.84	−4.52 ± 1.01	>0.05	~
Standard deviation of SL	2.09 ± 0.12	2.12 ± 0.08	>0.05	~
*k* (homodyned K)	0.73 ± 0.08	0.84 ± 0.23	<0.001	∗∗
*μ* (homodyned K)	0.18 ± 0.1	0.28 ± 0.26	<0.001	∗∗
*h* (homodyned K)	0.58 ± 0.03	0.55 ± 0.08	<0.001	∗∗
*m* (Nakagami)	0.54 ± 0.06	0.67 ± 0.17	<0.001	∗∗
*Ω* (Nakagami)	408736.82 ± 134753.77	189811.2 ± 166031.05	<0.001	∗∗
*α* (Nakagami)	219.74 ± 55.23	119.24 ± 98.33	<0.001	∗∗
Contrast	2.51 ± 1.11	2.01 ± 1.02	<0.05	∗
Correlation	0.59 ± 0.06	0.61 ± 0.07	<0.05	∗
Energy	0.135 ± 0.09	0.18 ± 0.10	<0.05	∗
Homogeneity	0.67 ± 0.07	0.7 ± 0.08	<0.05	∗

**Table 2:** Feature values for benign and malignant cases and statistical significance of features in the ATL dataset.

Feature	Benign values	Malignant values	*p* value	Statistical significance
Mean of MBF	76.44 ± 18.55	77.71 ± 11.84	>0.05	~
Standard deviation of MBF	6.26 ± 1.51	6.53 ± 1.52	>0.05	~
Mean of INT	64.77 ± 14.01	64.11 ± 6.93	>0.05	~
Standard deviation of INT	13.32 ± 1.09	12.91 ± 0.54	>0.05	~
Mean of SL	−3.28 ± 1.5	−3.45 ± 0.69	>0.05	~
Standard deviation of SL	1.73 ± 0.14	1.73 ± 0.09	>0.05	~
*k* (homodyned K)	0.35 ± 0.14	0.5 ± 0.1	<0.001	∗∗
*μ* (homodyned K)	0.16 ± 0.13	0.26 ± 0.21	<0.05	∗
*h* (homodyned K)	0.75 ± 0.08	0.67 ± 0.04	<0.001	∗∗
*m* (Nakagami)	0.33 ± 0.09	0.44 ± 0.09	<0.001	∗∗
*Ω* (Nakagami)	5116.67 ± 6622.77	1692.06 ± 997.2082	<0.05	∗
*α* (Nakagami)	31.21 ± 16.11	16.46 ± 6.6	<0.001	∗∗
Contrast	3.55 ± 1.64	2.97 ± 0.8	>0.05	~
Correlation	0.4 ± 0.07	0.38 ± 0.04	>0.05	~
Energy	0.17 ± 0.06	0.17 ± 0.07	>0.05	~
Homogeneity	0.66 ± 0.06	0.67 ± 0.05	>0.05	~

**Table 3:** Classification performance of the four selected features on the testing portion of the OASBUD dataset.

Classifier	Classification accuracy	Sensitivity	Specificity	AUC	95% CI
KNN	92.5%	95%	90%	0.963	0.823~0.997
SVM	87.5%	85%	90%	0.968	0.878~0.995
RF	95%	95%	95%	0.959	0.797~0.993

**Table 4:** Classification performance of the four selected features in the ATL dataset without resampling.

Validation	Classifier	Classification accuracy	Sensitivity	Specificity	AUC	95% CI
10-fold CV	k-NN	79.23%	34.62%	90.38%	0.805	0.705~0.879
	SVM	84.62%	42.31%	95.2%	0.895	0.803~0.946
	RF	85.38%	65.38%	90.38%	0.849	0.748~0.92
LOOCV	k-NN	78.462%	30.77%	90.38%	0.855	0.753~0.918
	SVM	84.62%	42.31%	95.2%	0.892	0.811~0.944
	RF	87.3%	53.84%	92.3%	0.856	0.758~0.916

**Table 5:** Classification performance of the four selected features in the ATL dataset with SMOTE.

Validation	Classifier	Classification accuracy	Sensitivity	Specificity	AUC	95% CI
10-fold CV	k-NN	87.2%	94.23%	79.81%	0.948	0.895~0.966
	SVM	82.21%	82.69%	81.73%	0.909	0.857~0.942
	RF	87.98%	92.31%	83.68%	0.956	0.903~0.972
LOOCV	k-NN	88.94%	82.69%	95.2%	0.959	0.921~0.982
	SVM	82.69%	82.69%	82.69%	0.909	0.859~0.942
	RF	89.42%	88.46%	90.38%	0.948	0.903~0.971

**Table 6:** Classification performance of the four selected features in the ATL dataset with SMOTE-Tomek.

Validation	Classifier	Classification accuracy	Sensitivity	Specificity	AUC	95% CI
10-fold CV	k-NN	88.17%	93.55%	82.8%	0.943	0.90~0.97
	SVM	80.65%	80.65%	80.65%	0.909	0.858~0.947
	RF	93.01%	94.62%	91.4%	0.966	0.928~0.984
LOOCV	k-NN	86.6%	93.55%	79.57%	0.955	0.917~0.979
	SVM	84.95%	83.87%	86.02%	0.917	0.856~0.95
	RF	91.4%	93.55%	89.25%	0.964	0.93~0.985

**Table 7:** Comparison of classification performance of existing multiparametric QUS methods for breast lesion characterization and performance parameters obtained in this study.

	Parameters used	Classification accuracy	Sensitivity	Specificity	AUC
Hsu et al. [55]	Standard deviation of shortest distance (SS), contrast, and Nakagami *m*	89.4%	92.5%	86.3%	0.96
Klimonda et al. [28]	Contrast, correlation, energy, and homogeneity	91%	93%	88%	0.94
This study	Homodyned *k*, homodyned *h*, Nakagami *m*, and Nakagami *Ω*	93.01%	94.62%	91.4%	0.966

## Data Availability

The OASBUD dataset is publicly available via the Zenodo repository (10.5281/zenodo.545928), while the ATL dataset can be obtained through the corresponding author upon reasonable request.
